The article "IOT-Based Medical Informatics Farming System with Predictive Data Analytics Using Supervised Machine Learning Algorithms" was published in 2022. Journal: Comput Math Methods Med.

# IOT-Based Medical Informatics Farming System with Predictive Data Analytics Using Supervised Machine Learning Algorithms

**DOI:** 10.1155/2022/8434966

**Published:** 2022-08-30

**Authors:** Ashay Rokade, Manwinder Singh, Sandeep Kumar Arora, Eric Nizeyimana

**Affiliations:** ^1^School of Electronics and Electrical Engineering, Lovely Professional University, Punjab, India; ^2^College of Science and Technology, University of Rwanda, Rwanda

## Abstract

In the farming industry, the Internet of Things (IoT) is crucial for boosting utility. Innovative agriculture practices and medical informatics have the potential to increase crop yield while using the same amount of input. Individuals can benefit from the Internet of Things in various ways. The intelligent farms require the creation of an IoT-based infrastructure based on sensors, actuators, embedded systems, and a network connection. The agriculture sector will gain new advantages from machine learning and IoT data analytics in terms of improving crop output quantity and quality to fulfill rising food demand. This paper described an intelligent medical informatics farming system with predictive data analytics on sensing parameters, utilizing a supervised machine learning approach in an intelligent agricultural system. The four essential components of the proposed approach are the cloud layer, fog layer, edge layer, and sensor layer. The primary goal is to enhance production and provide organic farming by adjusting farming conditions as per plant needs that are considered in experimentation. The use of machine learning on acquired sensor data from a prototype embedded model is investigated for regulating the actuators in the system. Then, an analytics and decision-making system was built at the fog layer, employing two supervised machine learning approaches including classification and regression algorithms using a support vector machine (SVM) and artificial neural network (ANN) for effective computation over the cloud layer. The experimental results are evaluated and analyzed in MATLAB software, and it is found that the classification accuracy using SVM is much better as compared to ANN and other state of art methods.

## 1. Introduction

Data gathering and using data to inform practical farming decisions is undergoing a significant agricultural revolution. Intelligent culture is the request of modern news and ideas of technology (ICT) in farming, to degree machine intelligence algorithms, and the rationalization of raw material use, as a capital-located system and state-of-the-art electronics in drink farming in tenable and environmentally intimate habits. Innovative technologies are helping the plurality of people everywhere the experience in a type of ways. The Internet of Things (IoT) and dossier data, such as grown dossier data and data learning, are immediately playing a more and more critical duty in people's everyday lives, admitting them to change their environment more surely [1–3]. In general, IoTs and data reasoning are secondhand in the agromodern and environmental subdivisions for two together diagnostics and control of brilliant culture arrangements, to provide essential facts to the final laborer and services about the footing and properties of agroproduction and structures [4–6].  Figure 1 shows the overview of IoT-based smart agriculture factors.

Machine learning is being used to regulate actuators' intelligence. The algorithm uses data acquired about the plants' climatological and soil conditions to advise the farmer on what should be done efficiently. IoT is also utilized to collect sensor data from the field so that the data and ML algorithm recommendations may be made available on a UI platform, making it easier to keep track of the field in real time. In intelligent farming, supervised machine intelligence algorithms are used to create predictions on dossier acquired by sensors and to deliver agriculture solutions. The utilization of IoT devices gives an automatic data prediction solution. The obtained results will assist the farmer in making an informed decision [6, 7]. The proposed technology will boost system efficiency and forecast superior intelligence control options. The plant's growth will be affected by changing climatic circumstances in agriculture, resulting in a lower yield after the cultivation. As a result, environmental sensing parameters such as greenhouse gases, temperature, soil moisture, and light must all be maintained and monitored. This issue could be solved by implementing an Internet of Things (IoT) innovation in intelligent agriculture, which entails the precise application of certain greenhouse factors for optimal plant development, such as temperature management, water flow control, and light radiation, among other things [8, 9]. The main contributions of the paper are as follows.

- Develop efficient analytics and decision-making model which can be used for precise and intelligent farming using supervised machine learning
- Design of a four-layer framework for IoT-based intelligent farming system that can support the deployment of the low-cost farming system with intelligent solutions
- Presented a case study on adoption of IoT and data analytics on two greenhouse plants, Gerbera and Broccoli
- Evaluate the proposed analytics and decision-making model based on supervised machine learning performances through different experiment

The rest of the paper is organized as follows: In Section 2, the related work regarding intelligent model using various data analytic algorithms is discussed. The details of proposed intelligent farming framework are presented in Section 3.  Section 4 describes an experimental evaluation with results.  Section 5 finally presented conclusions towards proposed scheme.

## 2. Literature Review

Several researchers have developed an intelligent agriculture system with predictive intelligence for various applications. The summaries of those papers are listed below.

Suma [5] gives a survey of predicting analysis, Internet of Things (IoT) designs accompanying cloud presidency, and security wholes for multibreeding in the farming area, all while taking into account farmers' previous experiences. It also emphasizes the difficulties and issues that might be expected when incorporating contemporary technologies into traditional farming practices. For adequate decision support in IoT-based intelligent farming systems, Rezk et al. [6] propose an IoT-located intelligent production system linked with an effective prediction means called WPART established machine intelligence techniques to think crop productivity and dryness. Araby et al. [7] used a sensor network to collect field data from a variety of crops (potatoes, tomatoes, and so on). They before shipped the dossier to a machine-education invention to produce a warning meaning before effecting both the dossier and the warning communication by way of a graphical user interface (GUI). Several machine learning techniques have been built by Tageldin et al. [8] to predict plant infestation with CLW. The current research established a framework for machine learning to forecast CLW infestation in greenhouse plants. Aliar et al. [9] present a complete analysis of the various intelligent farming methods and architectures. It also examines various designs in depth and suggests acceptable solutions to today's intelligent farming issues. Sethy et al. [10] projected an arrangement that uses deep knowledge and IoT to monitor paddy fields by chance. The VGG16 preprepared network is being surveyed for paddy leaf ailment discovery and nitrogen rank belief. Kaushik et al. [11] propose an intelligent agriculture method that monitors the agricultural field and can help farmers increase productivity significantly. Siddiquee et al. [12] projected an IoT-based creative agriculture listening system accompanying different algorithms for discovery, quantification, adulthood testing, and diseased produce detection.

Nourelhouda et al. [13] developed and deployed a ground-breaking wireless mobile robot that uses the Internet of Things (IoT) to conduct a range of outdoor chores. More precise and efficient data, as well as a reduction in the workforce, are among the benefits of this endeavor. Sekaran et al. [14] grew a structural foundation that integrates the Internet of things (IoT) accompanying crop results, utilizing cloud estimating to monitor crops using different measures and orders. The procedure supplies a certain-time dossier study from sensors established in crops and produces a result for the grower, which is necessary for crop progress listening and saves the grower's time and strength. The concept of security and privacy in cloud computing can be implemented to design prototype for cloud layer devices [15–17]. and the demonstration of space time coding for MDL mitigation and capacity enhancement of FTS gives right direction for transmission criteria [18–20].

Kaur et al. [21] specify a scheme for capably monitoring and ruling abundant crop progress and result in limits. The system also engages machine intelligence and the Internet of Things (IoT) to predict crop yield. Liu [22] integrates the needs of knowledgeable agriculture complete happening to create an inventive farming floor based on Internet of Things electronics and machine intelligence, in addition to designing experiments to verify the policy's acting. Sharma et al. [23] grew a strategy that may be used to boost livestock productivity by predicting reproductive patterns, detecting consuming problems, and envisioning cow behavior using machine intelligence models and dossier from collar sensors, among other things. Lela Madhav and Sandeep [24] investigated a variety of machine learning algorithms, each with its own set of advantages and disadvantages ranging from the process to the final product. To get the most out of the model utilized, the user must first comprehend each model before implementing it to their application. Mekonnen et al. [25] provide a thorough examination of several machine learning algorithms in sensor data analytics in the agricultural environment. Perales Gómez et al. [26] detail a novel design for continuous land crop value listening established IoT and machine learning/deep learning technologies. Perales Gómez et al. [27] characterize an intelligent culture arrangement for crop production, namely, buxom on low-cost IoT sensors and common data storage and dossier science of logical analysis services connected to the Internet of Things Yang and Xu et al. [28] help and guide researchers in completely comprehending the strengths and potential drawbacks of deep learning in the horticultural sector. Cafuta et al. [29] present a whole replacement sensor dossier information with machine intelligence for plant well-being belief. Estimating plant strength admits for more comprehensive ebb periods and raises the nutritional content of the things produced. The fundamental goal of this case study, according to Bakthavatchalam et al. [30], is to evolve a model that forecasts extreme yield crops and precision farming. The projected method posing incorporates contemporary science, the Internet of Things, and farming's detracting measurements. Khalaf et al. [31] have given the efficiencies in cognitive radio enable 5G network which guarantees the use of 5G network to enhance system performance. Walia et al. [32] have emphasized on localization of dynamic wireless sensor networks. Singh et al. [33] give a brief idea about the energy-efficient cognitive body area network. Hassan et al. [34] proposed a survey for data sharing techniques for 5G. A. Rokade and Singh [35] give a brief analysis of intelligent farming techniques which helps us to propose a sustainable intelligent farming model. A. Kadu and Singh [36] emphasize on distinguish data analysis for telemedicine systems which describes the uses of IoT and machine learning. Hassan et al. [37–39] focus on the cognitive radio networks for improvement of capacity rate in 5G. Roy at el. [40] proposed a filter model for system enhancement. Moreover, the clustering technique can also be followed for the collection and aggregation of data, and data can be filtered through machine learning algorithms [41–46]. As part of the industry's technological progress, Teferaa et al. [47] emphasize emerging different automation approaches such as IoT, wireless communications, machine learning, artificial intelligence, and deep learning. Ha et al. [48] described a set of modern sensing applications that use machine learning-enabled intelligent sensor systems. In an intelligent greenhouse, Jin et al. [49] offer a bidirectional self-concentrating encoder-translator framework (BEDA) to build a seasoned prophet for numerous material limits with important nonlinearity and turbulence. Akhter et al. stated that [50] secondhand dossier data and machine intelligence in an IoT system to present an indicator model for Apple ailment in the sphere gardens of Kashmir basin. Quy et al. [51] judge the architecture (IoT designs, communication sciences, ample data conversion, and transform), applications, and research schedule of IoT-enabled brainy agriculture environments. The IoT ecosystem is described by Elijah et al. [52], who show how the integration of IoT and DA is enabling intelligent agriculture.

## 3. Methodology

### 3.1. Proposed Framework

The proposed intelligent farming system model for greenhouses is depicted in figure 2. The four basic architectural layers are the cloud layer, fog layer, edge layer, and sensor/device layer. The sensor layer includes the various sensors and actuators related to the field environment. The edge layer mainly consists of controller unit to which various sensors and actuators are interfaced for data acquisition and sending to fog layer for further process. The main objective of the fog layer is developing the analytics and decision-making model based on data acquired from the edge layer and provide the control signals to the edge layer for controlling of actuators. And finally, data representation of sensors and actuators is displayed on the cloud layer in the form of user interface (UI) dashboard. The suggested system is notable for its ability to assist farmers by providing greenhouse management using an IoT-based precision farming framework. The purpose is to supply agriculturists with remotely controlled greenhouse agricultural elements such as soil moisture, CO_2_, light, and temperature from afar, and depending on the soil moisture values, a controlling move for the greenhouse doors/windows to roll off/on may be made. Agriculturists are unable to visit the fields as a result of this physically.

#### 3.1.1. Sensor Layer

In this experiment, Gerbera and Broccoli are the crops that considered in the greenhouse, which is primarily a climate-sensitive environment. The sensors used to monitor factors in the greenhouse environment include a gas sensor, a dht11 sensor for temperature and humidity, a light sensor, a gas sensor, and a moisture sensor. Actuators will be chosen and deployed to control equipment such as fans and pumps by relaying parameters. Controlled RH, temperature, light, protection from rain, storms, and scorching sun, as well as pest and disease control, are all advantages of using a greenhouse management system for such a crop.

#### 3.1.2. Edge Layer

Sensors, known as nodes or edges, are put in the field at various locations and connected to a low-power microcontroller designed for IoT. We used a Node MCU ESP 32 in our experiment, which can gather and analyze data from sensors before transferring it to the edge layer's base station. Sensors must be calibrated and checked against an expected value to collect data in analog or digital form according to requirements. Data is collected for various climate variables, both healthy and unhealthy, to better comprehend all possible environmental situations and to assure crop survival through accurate crop management.

To test an intelligent greenhouse management system, a prototype experimental model was created using an embedded system device based on three primary layers that includes several sensors and a microprocessor at first layer, microcontrollers for a node at second layer, and cloud at third layer for data representation, as shown in Figure 3.

The proposed model tracks several greenhouse characteristics for two crops, Gerbera and Broccoli, in different climates. A microcontroller Node MCU ESP 32 is connected to all of the needed sensors for obtaining the greenhouse parameters. A personal computer collects data serially with timestamp values for data logging of various parameters. Temperature and humidity, which is taken from the DHT11 sensor, light intensity, which is taken from LDR sensor, CO_2_, which is taken from MQ2 sensor, and soil moisture, which is taken from Cu leads, are all continually monitored for ten days on the Adafruit IO cloud platform utilizing the MQTT protocol under day and night conditions within specific time intervals. Operational work flow of the proposed system is defined in Figure 4 in which four sensors are deployed at farm site with Node MCU ESP32 controller interfaced. The real-time data from sensors are monitored serially on personal computer through controller, and same data is sent on cloud.

#### 3.1.3. Fog Layer

The basic responsibility of the analytics and decision-making model is to control the actions at the edge layer and communicate the accompanying report to the cloud layer for the use of farmers. The in-charge order will create a machine intelligence treasure accompanying many processing states. The proposed methodology developed at the fog layer for data analytics system using machine learning algorithms typically classification modeling is as shown in Figure 5 and discussed in detail below.

At first, data from sensors is generated at the edge layer and then is acquired. Preprocessing of stored data is used to clean and correct the data. Data classification is based on its intended use by initializing the classifier, later after training of machine learning algorithms and validation of classifier so as to store trained classifier. Data was gathered by IoT devices, particularly sensors, which can collect data in real time or in small batches (temperature, humidity, camera vision, light intensity, etc.) (e.g., when to pump water). Decision-making based on predictions and data visualization through reports or dashboards were as follows: support vector machine (SVM) and multilayer perceptron neural network (MLP-ANN) are the two machine learning techniques that were primarily chosen for implementation. The advantages of selecting this algorithm are effective in high dimensional spaces and capability to learn nonlinear models.

Support vector machines (SVM) are a supervised classification and regression method. SVM's main idea is shifting nonlinear data to a new space for which the data may be separated linearly by employing a hyperplane that accurately separates the data by following two important conditions: because distinct classes of vectors will have various aspects, the distances between the hyperplane and the vectors must be used. The assumption function f has the following definition:

(1) $$\begin{array}{c} f\left(x_{i}\right)=\left\{{}_{-1\;\text{if}\;w.x\;+\;b\;<0}^{+1\;\text{if }w.x\;+\;b\geq 0}\right\}. \end{array}$$

Class +1 will be filling a place points above or on the hyperplane; when in fact, class -1 will be filling a place points beneath the hyperplane.

An artificial neural network (ANN) with one or more hidden layers is known as a Multilayer perceptron neural network. A perceptron is an interconnected system amounting to just an individual affecting the animate nerve organs model. It simulates high nonlinear functions, which are the foundation for deep learning neural networks. The degree of inaccuracy in an output node *j* in the nth data point (training example) can be represented by

(2) $$\begin{array}{c} e_{j}\left(n\right)=d_{j}\left(n\right)-y_{j}\left(n\right), \end{array}$$

where “*d*” is the goal value, and “*y*” is the perceptron's output value. The node weights can then be modified depending on adjustments that reduce the overall output error, as determined by

(3) $$\begin{array}{c} \in \left(n\right)=\frac{1}{2}\underset{j}{\sum }e_{j}^{2}\left(n\right). \end{array}$$

The trouble of selecting a set of ideal hyperparameters for a model knowledge invention is famous as hyperparameter bringing into harmony or optimization. An energetic limit is a profit for a limit that is to say used to influence the education process. The gridiron search method is utilized, which is an ultimate fundamental form of hyperparameter bringing into harmony. We merely produce a model each reasonable combination of all of the energetic-limit principles provided, judge each model, and pick the construction that gives the best results utilizing this arrangement. Below is a writing of the method for energetic limit regulating the model.

**Step 1 .**

Define a machine learning model.

**Step 2 .**

For the selected approach, define the range of possible values for all hyperparameters.

**Step 3 .**

Define a sampling mechanism for hyperparameter values.

**Step 4 .**

Create a criterion for judging the model.

**Step 5 .**

Develop a crossvalidation technique for determining the system's efficiency.

#### 3.1.4. Cloud Layer

Data from each node in the edge layer, which is subsequently processed and controlled at the base station, will be visualized at the cloud layer using an Adafruit IO cloud platform; farmers can track crop cultivation progress using a graphical interface- (UI-) based application. Adafruit IO is a platform for visualizing, responding to, and interacting with sensor data. With the support of MQTT, the dossier is likewise observed private and secure. MQTT (Message Queue Telemetry Transport) is a TCP/IP-located inconsequential issue-contribute contract. MQTT employs a message broker to route messages between senders who send them and receivers who are interested in receiving them. Messages can be published and subscribed to using the same client. Each message is associated with a specific subject, for example, as shown in Figure 6, how temperature sensor data from a greenhouse system is sent.

## 4. Experimental Result and Discussion

The proposed experimental plan is implemented on a prototype that has been tested practically on two crops, Gerbera and Broccoli, for various conditions. The acquired dataset has feature attribute of CO_2_ gas level (ppm), soil moisture (percent), light intensity (lux), humidity (percent), and temperature (Celsius) with output attribute pump (on/off), ventilation fan (on/off), and amount of light (low/medium/high). The values of dataset are taken under various conditions for several days and one hour per day. The mean of each day reading for every sensor's attribute is as shown in Figures 7–11. The two primary phases of experimentation are the creation of basic model embedded systems for plant growth and feeding, the construction of a sensor net for intelligent greenhouse monitoring, and the automation of actuators using supervised machine learning algorithms. The analytics and decision-making model classification was done on a laptop with a 2.30 GHz Intel ™ Core ™ CPU, 8 GB RAM, and Windows 10 (64 bit) operating system, with no other processes running in the background. MATLAB IDE is used to program the intelligent model, statistics, and machine learning toolbox from MATLAB that was utilized as tools. A confusion matrix as performance metrics is used to evaluate the system performance. Also, the accuracy, sensitivity, specificity, and *F*-score for the classification model and RMSE for the regression model are calculated from confusion matrix parameters: true positive (TP), false positive (FP), true negative (TN), and false negative (FN).

(4) $$\begin{array}{c} \text{Accuracy}=\frac{\left(\text{TP}+\text{TN}\right)}{\text{TP}+\text{TN}+\text{FP}+\text{FN}},\\ \text{Sensitivity}=\frac{\text{TP}}{\text{TP}+\text{FN}},\\ \text{Specificity}=\frac{\text{TN}}{\text{TN}+\text{FP}},\\ F-\text{score}=2*\frac{\text{TP}}{2\text{TP}+\text{FP}+\text{FN}},\\ \text{RMSE}=\text{sqrt}\left(\frac{\text{sum}\left({\left({\text{predicted}}_{\text{label}}-{\text{actual}}_{\text{label}}\right)}^{2}\right)}{\text{total}}\text{predictions}\right). \end{array}$$

The proposed approach employs an embedded system to analyze greenhouse execution parameters like as CO_2_, soil moisture, temperature, and plant light, yielding accurate results. All the readings are observed under several conditions and monitored on the personal computer over serial communication. All these sensor data are monitored over the Internet on the Adafruit IO cloud dashboard by publishing data from nodes to the broker of Adafruit. Then, the user can subscribe to this data to access it in real time.

The greenhouse doors/windows can also be rolled on/off depending on the soil moisture conditions. The plant photosynthesis process requires a high level of CO_2_ concentration and water in the evenings rather than during the day; with these two sources of energy, the photosynthesis method keeps the plant cool and encourages rapid growth. Because the greenhouse absorbs CO_2_ from day to night, it maintains a CO_2_ level maximum at night after completing a CO_2_ concentration level experiment in a greenhouse, as illustrated in Figure 6. As a result, as seen in Figure 6, the CO_2_ level decreases during the day.  Figure 7 depicts that moisture level of soil in wet and dry condition and accordingly motor turns on/off with amount of water. The environmental temperature and humidity are shown in Figures 8 and 9 inside and outside greenhouse; accordingly, and actuator fan or humidifier is controlled. The light intensity inside and outside greenhouse as shown in Figure 10 indicates that sufficient light is required for photosynthesis purpose; so, accordingly, artificial light is provided in accordance with it.

In the decision-making model, the confusion matrix for regression and classification model has been evaluated to get the desired result and calculate the different parameters such as accuracy, sensitivity, and latency after applying the proposed algorithms to the standard dataset. The two supervised machine learning models, SVM and MLP-ANN, were used to train and test the model using MATLAB software with statistics and machine learning toolbox. The both algorithms required best hyperparameters to train the model which are obtained by using the grid search CV algorithm which is mentioned in Table 1.

The simulation results for classification modeling are shown in Figures 12 and 13 mentioned below for the SVM and MLP algorithm, respectively. In these results, classification report results and confusion matrix for three output attributes pump, fan, and light are displayed. The performance of the classification model using confusion matrix is shown in Table 2. From this table, it is found that for all three output attributes, the SVM algorithm performed better as compared to MLP in all performance metrics; also, its graphical representation is as shown in Figure 14.

The simulation results for regression modeling are shown in Figures 15 and 16 mentioned below for the SVM and MLP algorithm, respectively. In these results, regression report results for three output attributes pump, fan, and light are displayed. The performance of the regression model using RMSE metric is shown in Table 3. From this table, it is found that for all three output attributes, the SVM regressor algorithm is performed better as compared to MLP regressor; also, its graphical representation is as shown in figure 17.

Finally, Table 4 shows the comparative analysis with the existing state of art methods. From the results, it is found that the proposed classification and regression model which is used for intelligent and precise smart farming for greenhouse model gives better results considering the classification model parameters using accuracy, sensitivity, specificity, and the regression model using RMSE.

## 5. Conclusion

This paper presented a machine learning-based smart farming system that makes use of IoT principles and capabilities. The suggested strategy can be applied in a smart agricultural setting where the decision-making model is supported by IoT-based systems. The data required for the analytics model is collected by using IoT-based embedded system device for two greenhouse plants with sensing parameters as input and related actuators as output. The two different analytics model is developed for intelligent and precise farming using classification and regression model. For both types of modeling, SVM and MLP are used. Finally, classification- and regression-based supervised machine learning algorithms are used to evaluate how well the smart farming system performs in intelligent and precise farming. The results demonstrated that SVM is perform better as compared to MLP and other existing state of art classification model. The suggested approach is also successful in creating smart agricultural systems with intelligent prediction-based decision support. On the basis of the experimental results, the proposed strategy also proved to be the most effective at providing actuators with predictions and control. Further, this proposed model can be used in real world scenario by making it robust and whether proof. Also, the analytics model will be varied as per the crop or plant consideration for certain scenario. The performance of the model can be improved by employing deep learning models with large dataset samples.

## Figures and Tables

**Figure 1:** Overview of an agriculture IoT [1].

**Figure 2:** Intelligent farming framework for greenhouse management.

**Figure 3:** Proposed framework for acquisition of data in the greenhouse environment.

**Figure 4:** Proposed experimental model.

**Figure 5:** Analytics and decision-making model.

**Figure 6:** Workflow of MQTT for sensor data.

**Figure 7:** Day and night time CO_2_ representation.

**Figure 8:** Dry and wet soil moisture representation.

**Figure 9:** Outside and inside greenhouse temperature representation.

**Figure 10:** Outside and inside greenhouse humidity representation.

**Figure 11:** Outside and inside greenhouse light intensity representation.

**Figure 12:** Classification approach result and confusion matrix MLP.

**Figure 13:** Classification approach result and confusion matrix SVM.

**Figure 14:** Performance of classification model.

**Figure 15:** Regression approach result for RMSE SVM.

**Figure 16:** Regression approach result for RMSE MLP.

**Figure 17:** Performance of the regression model.

**Algorithm 1:** Proposed algorithms.

**Table 1:** Hyperparameter tuning for classifier modeling.

Prediction algorithm	Model parameters	Range searched	Range selected
SVM classifier and regressor	Kernel max_iter	rbf, poly, sigmoid 10, 30, 50	Poly 10
MLP classifier and regressor	hidden_layer_size max_iter	10, 50, 100 100, 200, 300	100 200

**Table 2:** Performance evaluation of classification model.

Attributes	Accuracy (%)		Sensitivity (%)		Specificity (%)		*F*-score (%)	
	SVM	MLP	SVM	MLP	SVM	MLP	SVM	MLP
Pump	86.66	76.66	81.81	77.27	100	75	95.74	86.73
Light	96.66	70	100	89.47	90.90	36.36	95.95	73.91
Fan	90	83.33	94.11	82.35	84.61	84.61	89.88	86.41

**Table 3:** Performance evaluation of regression model.

Attributes	RMSE	
	SVM	MLP
Pump	0.0615	0.0074
Fan	0.0042	0.0020
Light	0.0256	0.0132

**Table 4:** Comparative analysis.

Ref	Accuracy (%)	Sensitivity (%)	Specificity (%)	*F*-score (%)	Latency (sec)	RMSE
[2]	—	93.59	94.63	96.30	—	—
[4]	—	—	—	—	—	0.2431
[6]	87.35	87.33	95.76	87.17	224.6	—
[7]	90	—	—	—	—	—
[13]	—	—	—	—	—	0.02726
Proposed work	91.10	91.97	91.83	92.1	6.49	0.0615

## Data Availability

The data will be availableupon request.
